The article "Mechanism Study of Cinnamomi Ramulus and Paris polyphylla Sm. Drug Pair in the Treatment of Adenomyosis by Network Pharmacology and Experimental Validation" was published in 2022. Journal: Evid Based Complement Alternat Med.

# Mechanism Study of Cinnamomi Ramulus and *Paris polyphylla* Sm. Drug Pair in the Treatment of Adenomyosis by Network Pharmacology and Experimental Validation

**DOI:** 10.1155/2022/2624434

**Published:** 2022-08-16

**Authors:** Keke Zhang, Zhou Zhou, Chuchu Wang, Mengdie Yu, Yiran Zhang, Yaxin Shi, Xin Wang, Yang Liu, Li Xu, Wei Shi, Zhiyong Liu

**Affiliations:** ^1^First Clinical Medical College, Shandong University of Traditional Chinese Medicine, Jinan, China; ^2^Shandong Provincial Hospital, Shandong First Medical University, Jinan, China; ^3^Affiliated Hospital of Shandong University of Traditional Chinese Medicine, Jinan, China

## Abstract

**Objective:**

To explore the molecular mechanism of the Cinnamomi ramulus and *Paris polyphylla* Sm. (C-P) drug pair in the treatment of adenomyosis (AM) based on network pharmacology and animal experiments.

**Methods:**

Via a network pharmacology strategy, a drug-component-target-disease network (D-C-T-D) and protein–protein interaction (PPI) network were constructed to explore the core components and key targets of C-P drug pair therapy for AM, and the core components and key targets were verified by molecular docking. Based on the results of network pharmacology, animal experiments were performed for further verification. The therapeutic effect of the C-P drug pair on uterine ectopic lesions was evaluated in a constructed AM rat model.

**Results:**

A total of 30 components and 45 corresponding targets of C-P in the treatment of AM were obtained through network pharmacology. In the D-C-T-D network and PPI network, 5 core components and 10 key targets were identified. Kyoto Encyclopedia of Genes and Genomes (KEGG) pathway enrichment analysis showed that the PI3K signaling pathway was the most significantly enriched nontumor pathway. Molecular docking showed that most of the core components and key targets docked completely. Animal experiments showed that the C-P drug pair significantly ameliorated the pathological changes of endometriotic lesions in AM model rats and inhibited PI3K and Akt gene expression, and PI3K and Akt protein phosphorylation. In addition, treatment with the C-P drug pair promoted AM cell apoptosis; upregulated the protein expression of Bax, Caspase-3, and cleaved Caspase-9; and restrained Bcl-2 expression.

**Conclusions:**

We propose that the pharmacological mechanism of the C-P drug pair in the treatment of AM is related to inhibition of the PI3K/Akt pathway and promotion of apoptosis in AM ectopic lesions.

## 1. Introduction

Adenomyosis (AM) is a gynecological disorder characterized by the abnormal appearance of endometrial glands and stroma in the myometrium. Increased dysmenorrhea, abnormal uterine bleeding (AUB), and infertility are the most typical symptoms of AM and severely affect the quality of life of patients [1]. Hormone therapy, which is often used as an effective palliative strategy, has side effects such as impaired ovarian reserve function, irregular vaginal bleeding, and infertility [2, 3]. Surgical hysterectomy, currently the only definitive treatment, is typically physiologically and psychologically traumatic for patients of reproductive age, but uterine-sparing surgery also has disadvantages: namely, removal of lesions is difficult and recurrence is common [4].

The article "Mechanism Study of Cinnamomi Ramulus and Paris polyphylla Sm. Drug Pair in the Treatment of Adenomyosis by Network Pharmacology and Experimental Validation" was published in 2022. Journal: Evid Based Complement Alternat Med.

Among alternative medicines, traditional Chinese medicine (TCM) has accumulated considerable clinical experience in AM treatment [5–7]. Cinnamomi ramulus (Guizhi), or branch of cinnamon, is believed in TCM to be able to relax muscles, warm the body and dredge meridians. Cinnamomi ramulus was first used for gynecological treatment in the formula Guizhi-Fuling Wan, as recorded in the Synopsis of the Golden Cabinet (Jin Gui Yao Lue), written by Zhang Zhongjing, and Cinnamomi ramulus is still used in clinics with remarkable effects [8, 9]. *Paris polyphylla* Sm. (Chonglou) is recorded in Shennong's Herbal Classic (Shen Nong Ben Cao Jing) and is believed to be able to relieve heat, remove toxic material, detumescence, and analgesic effects. Gongxuening capsules (Manufacturing Approval Number: Z20053256), which are commonly used in the clinical treatment of AM, are developed from *Paris polyphylla* Sm. and have been used to treat uterine diseases and blood stasis syndrome for decades [10–12].

In TCM treatment theory, prescriptions based on the concept of “drug pairs” can often achieve better results than individual drug prescriptions, as two drugs can often increase the effectiveness of each other. We extracted the monarch drugs (the drugs that play major roles in a formula), namely, Cinnamomi ramulus and *Paris polyphylla* Sm. (C-P), from Guizhi-Fuling Wan and Gongxuening capsules as a drug pair and explored their synergistic regulatory effects on an AM rat model in this study [13]. A previous study by our team demonstrated that when used in combination, Cinnamomi ramulus, *Paris polyphylla* Sm. and *Panax notoginseng* (Sanqi) reduced the levels of matrix metalloproteinases (MMP-2 and MMP-9), increased the expression of Bax and Caspase-3, and significantly reduced the proliferation and invasion ability of endometrial cells in AM model rats [14]. Using C-P drug pair is a promising therapeutic strategy for AM. However, the pharmacological mechanism of the C-P drug pair in the treatment of AM remains unclear.

TCMs are characterized by multiple components and multiple targets, which makes it difficult to further study the mechanism of the C-P drug pair in the treatment of AM. In recent years, the emergence of network pharmacology has provided an effective means to study the pharmacological mechanisms of TCMs. Construction and analysis of drug–component–target–disease (D-C-T-D) networks can enable the core components of TCMs and potential targets for disease treatment to be effectively discovered [15]. In this study, we used network pharmacology to construct D-C-T-D and protein–protein interaction (PPI) networks and searched for core components and key targets for C-P drug pairs to treat AM. Subsequently, we constructed a rat AM model to verify the network pharmacology results. Our findings provide a valuable reference for further study of the pharmacological mechanism of C-P in the treatment of AM.

The article "Mechanism Study of Cinnamomi Ramulus and Paris polyphylla Sm. Drug Pair in the Treatment of Adenomyosis by Network Pharmacology and Experimental Validation" was published in 2022. Journal: Evid Based Complement Alternat Med.

## 2. Materials and Methods

### 2.1. Acquisition of Active Components and Targets for the C-P Drug Pair

The ingredients and targets of Cinnamomi ramulus were obtained from the TCMSP database (https://old.tcmsp-e.com/index.php). The active ingredients obtained from the TCMSP database were screened under the conditions of oral bioavailability (OB) ≥30% and druglikeness (DL) ≥0.18, and the corresponding targets of the active ingredients were further obtained. The ingredients and corresponding targets of *Paris polyphylla* Sm. were obtained from the HERB database (https://herb.ac.cn/) and a literature search [16–22]. Standard name correction was performed for the obtained active ingredients using PubChem, and duplicate values were deleted. The SwissTargetPrediction database (https://www.swisstargetprediction.ch/) was used to predict the targets for the components obtained from the literature search [23, 24].

### 2.2. Search for AM-Related Targets

AM-related targets were searched in the GeneCards (https://www.genecards.org/), Coremine (https://coremine.com/medical/), and PharmGKB (https://www.pharmgkb.org/) databases using “Adenomyosis” as the retrieval keyword. The correlation score was used as a reference for each included target. The common targets between C-P and AM were identified using a Venn diagram.

### 2.3. Construction of the D-C-T-D Network

Microsoft Excel was used to determine the relationships among the drugs, active ingredients, common targets, and disease. The data were then imported into Cytoscape software, and a D-C-T-D network model was built. In the model, the nodes represent the herbs, components, targets, and disease, and edges represent relationships between two nodes. The number of associations of each node is used to calculate the “degree.”

### 2.4. Construction of the PPI Network and Screening of Key Targets

The overlapping targets between the C-P active ingredient targets and the AM-related targets were imported into the STRING database (https://www.string-db.org/cgi/input.pl), and “*Homo sapiens*” was used as the screening criterion to obtain the PPI relationship [25]. The results were then imported into Cytoscape 3.8.0 software to construct a PPI network of intersecting targets of the C-P drug pair and AM. The core targets were obtained by screening related targets according to the degree centrality (DC), betweenness centrality (BC), and closeness centrality (CC).

The article "Mechanism Study of Cinnamomi Ramulus and Paris polyphylla Sm. Drug Pair in the Treatment of Adenomyosis by Network Pharmacology and Experimental Validation" was published in 2022. Journal: Evid Based Complement Alternat Med.

### 2.5. Gene Ontology (GO) Biological Process and Kyoto Encyclopedia of Genes and Genomes (KEGG) Pathway Enrichment Analyses

DAVID 6.8 (https://david.ncifcrf.gov/) was utilized to perform GO biological process enrichment and KEGG pathway analysis on the overlapping targets between C-P and AM [26]. The top 20 KEGG pathways and the top 20 biological processes from GO analysis with the most significant enrichment were plotted.

### 2.6. Molecular Docking of Core Components and Key Targets

The five components with the highest degrees were identified as core components in the D-C-T-D network, and the 2D structures of the core components were downloaded from PubChem (https://pubchem.ncbi.nlm.nih.gov/) database. The 3D structures of key target proteins were downloaded from the RCSB database (https://www.rcsb.org/search). Chem3D software was used to preprocess the components, and AutoDock Vina software was used for molecular docking analysis of the core components and key targets. The binding energy between the component and the protein was used to assess the degree of binding. PyMOL software was used to visually display part of the structure.

### 2.7. Experimental Drugs

The herbal medicines were supplied by the Affiliated Hospital of Shandong University of Traditional Chinese Medicine (Jinan, China) and verified by Prof. Feng Li. Cinnamomi ramulus and *Paris polyphylla* Sm. were mixed at a standard ratio of 5 : 4 and were subjected to reflux extraction twice with 10 times the volume of distilled water for 1 h each. The extracts were then mixed thoroughly and concentrated to a relative density of 1.20–1.25 (70–80°C). The dosage of the C-P drug pair liquid used in subsequent animal studies was 2.7 g/kg/day. Mifepristone was purchased from Beijing Zizhu Pharmaceutical Co., Ltd. (National Medicine Standard H20010633). The final dosage was 1.25 mg/kg/day [27].

### 2.8. Reagents

Rabbit anti-Caspase-3 (bs-0081R) and Caspase-9 (bs-0049R) polyclonal antibodies were obtained from Beijing Bioss Biotechnology Co., Ltd. (Beijing, China). A Bax monoclonal antibody (60267-1-Ig) and a Bcl-2 polyclonal antibody (12789-1-AP) were obtained from Wuhan Proteintech Biotechnology Co., Ltd. (Wuhan, China). PI3 kinase p85 alpha (phospho-Y607, p-PI3K) (ab182651), GAPDH (EPR16891, loading control) (ab181602) and Akt (phospho-T308, p-Akt) (ab38449) antibodies were obtained from Abcam, Inc. (Cambridge, MA, USA).

The article "Mechanism Study of Cinnamomi Ramulus and Paris polyphylla Sm. Drug Pair in the Treatment of Adenomyosis by Network Pharmacology and Experimental Validation" was published in 2022. Journal: Evid Based Complement Alternat Med.

### 2.9. Experimental Grouping, Modeling, and Intervention

Forty female Wistar rats and 30 male Wistar rats purchased from Beijing Vital River Laboratory Animal Technology Co., Ltd., were housed in the SPF Animal Experimental Center of the Affiliated Hospital of Shandong University of Traditional Chinese Medicine. All rats had free access to a commercial diet and tap water. All the experimental procedures conformed to the regulations described in the Guide to the Care and Use of Laboratory Animals of the USA National Institutes of Health. The ethical review was approved by the Affiliated Hospital of Shandong University of Traditional Chinese Medicine (AWE-2019-009). According to the random number table method, 40 female Wistar rats were divided as follows: 10 mice served as the blank group, and the remaining 30 were prepared for modeling. Animal models were established according to previous studies [28]. The pituitary gland of male rats was implanted into the uterine cavity of female rats, and 800,000 U of penicillin was injected for a week to prevent infection. Three months later, female rats were randomly divided into the model group, C-P group, and positive control group. According to the “Equivalent Dose Table for Conversion of Human and Animal Body Surface Areas,” the rats were administered normal saline, C-P drug pair liquid, and mifepristone by gavage. After 30 days of treatment, the rats were euthanized by cervical dislocation, and their uterine tissues were collected.

### 2.10. Pathological Observation

The uterine tissues were fixed in 4% paraformaldehyde solution and embedded in paraffin, and 5 *μ*m-thick sections were prepared for hematoxylin and eosin (H&E) staining. All images were acquired using a NanoZoomer S60 Digital slide scanner (Hamamatsu, Japan).

### 2.11. Immunohistochemistry

Bax, Bcl-2, Caspase-3, and Caspase-9 protein expressions in uterine tissues were detected using the immunohistochemistry streptavidin-peroxidase (SP) method. The regions were randomly selected under the microscope, and the cumulative optical density, area, and average density of the regions were measured using ImageJ (version 1.8.0).

### 2.12. Real-Time PCR

The expression of genes was quantified using the real-time PCR ΔΔCT method with a LightCycler 480II platform (Roche, Switzerland). Total RNA was purified using a Simply P Total RNA Extraction Kit according to the manufacturer's instructions. cDNA was synthesized with a ReverTra Ace qPCR RT Kit. Quantitative PCR was performed using a LightCycler 480II Real-Time PCR Detection System. All primers were synthesized by Integrated DNA Technology (BioSune, China). The primer sequences for mRNA analysis were as follows: phosphatidylinositol 4,5-bisphosphate 3-kinase catalytic subunit alpha isoform (PIK3CA) forward 5′-CTGCAGTTCAACAGCCACAC-3′ and reverse 5′-CCAGCTGCCATCTCAGTTCA-3′; Akt1 forward 5′-AAGGTTTGCTGGGTGAGTGA-3′ and reverse 5′-CTCCTCAGGCGTTTCCACAT-3′. GAPDH expression was used to normalize gene expression.

The article "Mechanism Study of Cinnamomi Ramulus and Paris polyphylla Sm. Drug Pair in the Treatment of Adenomyosis by Network Pharmacology and Experimental Validation" was published in 2022. Journal: Evid Based Complement Alternat Med.

### 2.13. Western Blotting

Uterine tissues (50 mg) collected from each group were homogenized and lysed in RIPA lysis buffer and then analyzed to detect the protein concentration using a BCA kit. Tissue total proteins were loaded onto 10% SDS–PAGE gels and transferred onto a PVDF membrane. The membrane was blocked using 5% skim milk and then incubated overnight with primary antibodies (p-PI3K, p-Akt, Bax, Bcl-2, and Caspase-9) at 4°C. The membrane was then incubated with a secondary antibody. Western blot analysis was performed using a ChemiDoc Imaging System (BIO-RAD, USA). The density of the signal was quantified by ImageJ.

### 2.14. Statistical Analyses

All data were analyzed using GraphPad Prism 8 (version 8.0.2) and are expressed as the mean ± standard deviation (SD). Comparisons between two groups were performed using Student's *t*-tests, whereas the significance of differences among three or more experimental groups was determined by one-way analysis of variance. A value of *P* < 0.05 was considered to indicate statistical significance. Diagrams were drawn using GraphPad Prism 8.

## 3. Results

### 3.1. Acquisition of Active Components and Targets for the C-P Drug Pair

A total of six active components and 50 corresponding targets of Cinnamomi ramulus were obtained from the TCMSP database. A total of 24 active components of *Paris polyphylla* Sm. were obtained from the HERB database and a literature search, and 360 targets corresponding to the active components of *Paris polyphylla* Sm. were obtained. A total of 384 potential targets of the C-P drug pair were identified after removing the repetition. A total of 504 targets related to AM were obtained through database retrieval. A Venn diagram revealed 45 intersecting targets between the C-P drug pair and AM (Figure 1(a)).

### 3.2. Construction of the D-C-T-D Network

Two herbs, 30 components, 45 targets, and 1 disease were classified and imported into Cytoscape 3.8.0 software to draw the D-C-T-D network (Figure 1(b)), which was composed of 77 nodes and 208 edges. “Degree” refers to the number of connections between each node and other nodes. Components in the network were screened according to a degree. The top five nodes based on the number of degrees were as follows: ecdysone (degree = 17), pinnatasterone (degree = 14), 20-hydroxyecdysone (degree = 14), flavone (degree = 12), and diosgenin (degree = 9). These molecules are thought to be the core components of the C-P drug pair in the treatment of AM (Table 1).

The article "Mechanism Study of Cinnamomi Ramulus and Paris polyphylla Sm. Drug Pair in the Treatment of Adenomyosis by Network Pharmacology and Experimental Validation" was published in 2022. Journal: Evid Based Complement Alternat Med.

### 3.3. Construction of the PPI Network and Screening of Key Targets

Forty-five common targets were imported into the STRING database to obtain the PPI relationship data, which were imported into Cytoscape 3.8.0 software to construct the PPI network (Figure 2(a)). Finally, the first ten targets were selected as the key targets for C-P in the treatment of AM according to the BC, CC, and DC (Figure 2(b)). The key targets included PIK3CA, interleukin-8 (CXCL8), interleukin-6 (IL6), estrogen receptor (ESR1), cellular tumor antigen p53 (TP53), c-c motif chemokine 2 (CCL2), vascular endothelial growth factor A (VEGFA), fibroblast growth factor 2 (FGF2), prostaglandin G/H synthase 2 (PTGS2), and interleukin-10 (IL10) (Table 2).

### 3.4. GO Biological Process and KEGG Pathway Enrichment Analyses

We used the DAVID database to conduct an enrichment analysis of GO and KEGG pathways for the intersected targets of the C-P drug pair and AM and obtained a total of 327 biological processes (BPs) and 118 signaling pathways with a *P* value <0.05 as screening conditions. R 4.0.2 software and its expansion package were used to draw bubble charts to show the top 20 significantly enriched BP and KEGG terms (Figure 3(a), 3(b)). The results of KEGG pathway enrichment showed that the PI3K-Akt signaling pathway was the most significant non-tumor-related pathway. In the GO analysis results, phosphorylation regulation of the PI3K signal and positive regulation of protein phosphorylation were also significantly enriched. In addition, PIK3CA, the core protein of the PI3K-Akt signaling pathway, was a key target in the PPI network screening. Therefore, we concluded that the PI3K-Akt signaling pathway plays a key role in the C-P treatment of AM. This conclusion was verified in the animal experiments performed for this study.

### 3.5. Verification of Molecular Docking

The 2D structures of the five core components in the D-C-T-D network were obtained from the PubChem database. The 3D structures of 10 key targets in the PPI network were obtained from the RCSB database. Five core components and 10 targets were docked. Binding energy was used to evaluate the degree of binding of ingredients to proteins, and a binding energy <−5 kcal/mol was considered to indicate that component and target could bind. The results of our study showed that the core components had good overall docking with the key targets (Figure 4(a)), indicating that these components may play a role in the treatment of AM by acting on the key targets. We used PyMOL to demonstrate some of the well-matched results (Figure 4(b)–4(g)). The blue lines between molecules represent hydrogen bonds and the yellow lines represent hydrophobic interactions.

The article "Mechanism Study of Cinnamomi Ramulus and Paris polyphylla Sm. Drug Pair in the Treatment of Adenomyosis by Network Pharmacology and Experimental Validation" was published in 2022. Journal: Evid Based Complement Alternat Med.

### 3.6. H&E Staining of Uterine Tissue

In the control group, the uterine morphology was intact and the muscular layer was continuous. The boundary between the muscular layer and the endometrium was clear, and no gland or endometrium tissue invasion was observed. However, the muscle layer in the model group was thickened with gland invasion and the boundary was blurred. Compared with that in the model group, the muscle layers in the C-P and mifepristone groups were almost intact. The boundary between the muscle layer and the intima layer was fairly clear, and fewer glands invaded the muscle layer (Figure 5)(a).

### 3.7. Effect of the C-P Drug Pair on the PI3K-Akt Signaling Pathway

The results of real-time PCR analysis indicated that PIK3CA and Akt1 mRNA expression was significantly higher in the AM model group than in the control group. The C-P drug pair and mifepristone significantly suppressed PIK3CA and Akt1 mRNA expression in AM rats compared with that in model rats (Figure 5(b), 5(c)). The expression trend of the P-PI3K and P-Akt proteins in Western blot analysis was the same as that observed with real-time PCR (Figure 6(a)).

### 3.8. The C-P Drug Pair Promoted Apoptosis in Ectopic Uterine Lesions

We observed changes in the apoptosis-related indicators Bax, Bcl-2, Caspase-3, and Caspase-9 in AM rats after C-P treatment based on tissue- and protein-level detection. The immunohistochemistry results showed that Bax (Figure 7(a)), Caspase-3 (Figure 7(c)) and Caspase-9 (Figure 7(d)) expression in the AM model group was significantly weaker than that in the control group, while Bcl-2 (Figure 7(b)) expression was stronger than that in the control group. Bax, Caspase-3, and Caspase-9 expressions were significantly enhanced in the C-P and mifepristone-treated AM groups than in the AM model group, while Bcl-2 expression was attenuated. The Western blot analysis results were consistent with the immunohistochemistry results. Compared with that in the control group, Bax and C-Caspase-9 protein expression in the model group was significantly reduced, and Bcl-2 protein expression was significantly induced. Compared with that in the model group, Bax and C-Caspase-9 protein expression in the C-P group and mifepristone group was significantly increased, whereas Bcl-2 protein expression was significantly suppressed. However, no significant difference in Caspase-9 expression was noted between groups, suggesting that C-P might promote Caspase-9 activation (Figure 6(b)).

The article "Mechanism Study of Cinnamomi Ramulus and Paris polyphylla Sm. Drug Pair in the Treatment of Adenomyosis by Network Pharmacology and Experimental Validation" was published in 2022. Journal: Evid Based Complement Alternat Med.

## 4. Discussion

Although AM is a condition of benign gynecological lesions, the lesions show abnormal tumor characteristics including endometrial cell proliferation, apoptosis, invasion, and migration. Compared with radical hysterectomy, TCM treatment has positive effects on women's fertility. Cinnamomi ramulus and *Paris polyphylla* Sm. are commonly used in TCM [29–31]. The pathological basis of AM in the theory of TCM is that the blood of the meridian in the uterus is cold and stagnant. In TCM, it is believed that Cinnamomi ramulus can warm the meridian and promote blood circulation and that *Paris polyphylla* Sm. can remove blood stasis. Cinnamomi ramulus and *Paris polyphylla* Sm. are commonly used to warm meridians, remove blood stasis and relieve pain.

Modern pharmacological studies have shown that the active components of Cinnamomi ramulus can inhibit the activity, migration, and glycolysis of endometrial stromal cells by inhibiting pyruvate kinase PKM (PKM2) transcription induced by the NF-*κ*B signaling pathway [32]. *Paris polyphylla* Sm. and its derivatives have been widely used to treat abnormal endometrial bleeding [11]. *Paris polyphylla* Sm. is also rich in a variety of saponins that have been widely used to combat abnormal cell proliferation and migration and to promote apoptosis of abnormal cells [33, 34].

TCM is characterized by the use of multiple drugs with multiple components and targets for the treatment of diseases. This complexity can hinder the exploration of the molecular mechanisms of TCM drugs in the treatment of AM from the perspective of precision medicine. Network pharmacology is useful for constructing D-C-T-D networks and PPI networks of drug–disease intersection targets based on the abovementioned characteristics of TCM. Through network analysis, the core components and key targets of TCM in the treatment of diseases can be obtained. This research method is beneficial for precision research on TCM and provides an effective means for identifying new targets for disease treatment.

In our study, a total of 30 components and 45 corresponding targets of the C-P drug pair related to AM were obtained through network pharmacology. In the D-C-T-C network, ecdysone, pinnatasterone, 20-hydroxyecdysone, flavone and diosgenin exhibited high degree numbers. These results suggest that these compounds may play a major role in the pharmacological mechanism of C-P in the treatment of AM. 20-Hydroxyecdysone has been reported to be a natural active component with the potential to promote apoptosis and autophagy in cancer cells [35]. In addition, as a natural steroid saponin, diosgenin can promote apoptosis of abnormally proliferating endometrial cells by regulating the apoptosis-related proteins Bcl-2, Caspase3, and Caspase9 [36]. Secretory dysfunction of the ovaries is considered to be an important factor affecting AM [37]. The synthesis of ecdysone in humans is regulated by the estrogen receptor (ER) [38]. Studies have shown that exogenous supplementation of ecdysone in ovariectomized female mice can inhibit a variety of metabolic diseases caused by the ovarian loss [39, 40].

The article "Mechanism Study of Cinnamomi Ramulus and Paris polyphylla Sm. Drug Pair in the Treatment of Adenomyosis by Network Pharmacology and Experimental Validation" was published in 2022. Journal: Evid Based Complement Alternat Med.

Through analysis of the PPI network, we obtained 10 potential core targets of C-P therapy for AM: PIK3CA, IL10, IL6, ESR1, CCL2, TP53, VEGFA, FGF2, PTGS2, and CXCL8. PIK3CA is the catalytic subunit of the dimeric protein PI3K. As the core mediator of the PI3K signaling pathway, PI3K is a critical mediator of cell survival, and its downstream MTOR protein is an important protein involved in autophagy to avoid apoptosis [41]. IL6 and VEGFA are involved in inflammation and abnormal angiogenesis in AM, respectively [42, 43]. ESR1, a receptor protein of estrogen, is involved in the balance of estrogen in women, and studies have shown that disruption of this balance is an important factor in the occurrence and progression of AM [44]. IL10 is one of the major anti-inflammatory cytokines, and abnormal expression of IL10 in AM may impair endometrial receptivity and thus affect embryo implantation [45]. In summary, multiple core targets obtained through PPI network analysis play important roles in the pathological process of AM.

Through KEGG enrichment analysis of overlapping C-P and AM targets, we found that the PI3K signaling pathway was the most significant nontumor pathway, and GO enrichment analysis showed that phosphorylation (activation) of the PI3K signaling pathway was a significantly enriched biological process. In the molecular docking results, PIK3CA (PI3K) was able to dock with multiple core components. Therefore, PIK3CA may represent an important target of C-P in the treatment of AM. Previous studies have demonstrated that PI3K-Akt activation in AMs promotes endometrial cell proliferation [46]. In addition, PI3K and Akt gene and protein expression are upregulated in AM patients compared with controls without endometrial lesions [47]. The most widely studied PI3K is a heterodimer composed of a regulatory subunit (P85) and a catalytic subunit (PIK3CA, PIK3CB, PIK3CD, and PIK3CG). To generate the active form of PI3K, the phosphorylation sites in the SH2 and SH3 domains of the P85 subunit bind to the corresponding binding proteins, and phosphorylation occurs. Phosphorylated PI3K also activates the downstream protein Akt through phosphorylation and ultimately regulates a variety of biological pathways. In this study, we assessed the status of the PI3K/Akt signaling pathway by detecting P-PI3K and P-Akt protein levels. The PI3K/Akt pathway was activated in the AM model group compared with the control group, whereas PI3K and Akt phosphorylation was inhibited after C-P intervention.

The article "Mechanism Study of Cinnamomi Ramulus and Paris polyphylla Sm. Drug Pair in the Treatment of Adenomyosis by Network Pharmacology and Experimental Validation" was published in 2022. Journal: Evid Based Complement Alternat Med.

The PI3K/Akt signaling pathway is closely related to Bcl-2 family proteins. When stimulated, active Akt leads to the phosphorylation of the proapoptotic protein Bad and inhibits the translocation of Bad from the cytoplasm to the mitochondria, thereby inhibiting mitochondrial dysfunction. Mitochondrial dysfunction stimulates downstream Caspase-3 and Caspase-9. The cleaved forms of Caspase-3 and Caspase-9 regulate other protein substrates, ultimately triggering apoptosis [48]. Moreover, the PI3K/Akt pathway mediates apoptosis in many gynecological diseases. PI3K/Akt is involved in uterine leiomyoma apoptosis and proliferation [49, 50]. Naringenin increases apoptosis of human endometriosis cells through the inactivation of the PI3K pathway [51]. CD47 overexpression activates the PI3K/Akt/mTOR signaling pathway in endometrial carcinoma cell lines to reduce cancer cell apoptosis [52]. In this study, through detection of apoptosis-related indicators, we found that the proapoptotic proteins Bax, Caspase-3, and Caspase-9 were significantly downregulated in the AM model group, whereas the antiapoptotic protein Bcl-2 was significantly upregulated. After C-P intervention, the Bax, Caspase-3, and Caspase-9 proteins were significantly upregulated, whereas Bcl-2 was significantly downregulated. In conclusion, the pharmacological mechanism by which C-P improves AM is related to the inhibition of the PI3K signaling pathway and the promotion of AM lesion cell apoptosis.

## 5. Conclusion

Network pharmacology and animal experiments showed that the C-P drug pair can significantly delay disease progression in AM rats. We propose that the pharmacological mechanism of C-P in the treatment of AM is related to inhibition of the PI3K pathway and promotion of apoptosis in AM ectopic lesions. However, unfortunately, the pharmacological components of C-P are not well characterized, and whether C-P regulates apoptosis through the PI3K/Akt pathway remains unclear. We will further explore the effective components and pharmacological mechanism of C-P in the treatment of AM through subsequent experiments.

## Figures and Tables

**Figure 1:** Venn diagram and drug-active component-target-disease network. (a) The Venn diagram shows 45 overlapping targets between AM-related targets and active compound-related targets. (b) Drug-component-target-disease (D-C-T-D) network of C-P in the treatment of AM. The blue nodes represent drugs, the yellow nodes represent active components, the dark green nodes represent targets, and the red nodes represent disease.

The article "Mechanism Study of Cinnamomi Ramulus and Paris polyphylla Sm. Drug Pair in the Treatment of Adenomyosis by Network Pharmacology and Experimental Validation" was published in 2022. Journal: Evid Based Complement Alternat Med.

**Figure 2:** PPI network and core targets. (a) PPI network of potential C-P therapeutic targets for AM. (b) 10 core targets in the PPI network.

**Figure 3:** Bubble charts. (a) Bubble chart for GO enrichment analysis. (b) Bubble chart for KEGG enrichment analysis. The closer the bubble color is to red, the smaller the *P* value is, and the bubble size reflects the number of enriched genes.

**Figure 4:** Results of molecular docking. (a) Heatmap of binding energy. Unit: kcal/mol. (b) Molecular docking of PIK3CA with 20-hydroxyecdysone. (c) Molecular docking of PIK3CA with diosgenin. (d) Molecular docking of PIK3CA with ecdysone. (e) Molecular docking of PIK3CA with pinnatasterone. (f) Molecular docking of PIK3CA with flavone. (g) Molecular docking of PTGS2 with diosgenin.

**Figure 5:** H&E staining and results of real-time PCR. (a) H&E staining. (b)The mRNA expression of PIK3CA and Akt1 (compared with control group, ^*∗*^*P* < 0.05, ^*∗∗*^*P* < 0.01, ^*∗∗∗*^*P* < 0.001. Compared with model group, ^#^*P* < 0.05, ^##^*P* < 0.01, ^###^*P* < 0.001).

**Figure 6:** Results of western blotting assays. (a) The expression of p-PI3K and p-Akt. (b) The expression of Bax, Bcl-2, Caspase-9 and C-Caspase-9 (compared with control group, ^*∗*^*P* < 0.05, ^*∗∗*^*P* < 0.01, ^*∗∗∗*^*P* < 0.001. Compared with model group, ^#^*P* < 0.05, ^##^*P* < 0.01, ^###^*P* < 0.001).

**Figure 7:** The results of immunohistochemistry. (a) Bax. (b) Bcl-2. (c) Caspase-3. (d) Caspase-9. (e) Quantitative analysis of immunohistochemistry (compared with control group, ^*∗*^*P* < 0.05, ^*∗∗*^*P* < 0.01, ^*∗∗∗*^*P* < 0.001. Compared with model group, ^#^*P* < 0.05, ^##^*P* < 0.01, ^###^*P* < 0.001).

**Table 1:** Core components.

Component name	PubChem CID	Molecular formula	Molecular weight	Degree
Ecdysone	19212	C27H44O6	464.6	17
Pinnatasterone	15214617	C27H44O7	480.6	14
20-Hydroxyecdysone	146158258	C33H52O7	560.8	14
Flavone	10680	C15H10O2	222.24	12
Diosgenin	99474	C27H42O3	414.6	9

**Table 2:** Information of the 10 key targets.

Gene	Degreecentrality	Betweennesscentrality	Closenesscentrality
TP53	18	0.189524	0.558442
VEGFA	17	0.15469	0.52439
PTGS2	13	0.117131	0.518072
ESR1	12	0.086981	0.477778
PIK3CA	9	0.068537	0.488636
IL6	15	0.063904	0.5375
CXCL8	12	0.048844	0.472527
FGF2	11	0.046362	0.43
CCL2	11	0.036549	0.457447
IL10	12	0.031854	0.467391

The article "Mechanism Study of Cinnamomi Ramulus and Paris polyphylla Sm. Drug Pair in the Treatment of Adenomyosis by Network Pharmacology and Experimental Validation" was published in 2022. Journal: Evid Based Complement Alternat Med.

## Data Availability

All datasets for this study are included in the manuscript, further inquiries can be directed to the corresponding authors.
